# Nogo-A Is a Potential Prognostic Marker for Spinal Cord Injury

**DOI:** 10.1155/2022/2141854

**Published:** 2022-05-04

**Authors:** Haojun Shi, Liangyu Xie, Wenchang Xu, Shengnan Cao, Yuanzhen Chen

**Affiliations:** ^1^Second Clinical Medical College of Henan University of Traditional Chinese Medicine, Zhengzhou, Henan, China; ^2^Bone Biomechanics Engineering Laboratory of Shandong Province, Neck-Shoulder and Lumbocrural Pain Hospital of Shandong First Medical University, Shandong First Medical University & Shandong Academy of Medical Sciences, Jinan, Shandong, China

## Abstract

**Objective:**

Spinal cord injury (SCI) has become prevalent worldwide in recent years, and its prognosis is poor and the pathological mechanism has not been fully elucidated. Nogo-A is one of the isoforms of the neurite outgrowth inhibitory protein reticulon 4. The purpose of this study was to determine whether Nogo-A could be used as a marker for predicting the prognosis of SCI.

**Methods:**

We screened eligible SCI patients and controls based on inclusion and exclusion criteria. We also collected baseline clinical information and peripheral venous blood of the enrolled population. Participants' baseline serum Nogo-A levels were measured by enzyme-linked immunosorbent assay (ELISA). The American Spinal Injury Association (ASIA) scale was used to evaluate the prognosis of SCI patients after 3 months.

**Results:**

Baseline clinical information (age; gender; smoking; drinking; SBP, systolic blood pressure; DBP, diastolic blood pressure; fasting blood glucose; WBC, white blood cells; CRP, C-reactive protein) of SCI patients and controls were not statistically significant academic differences (*p* > 0.05). The baseline serum Nogo-A levels of SCI patients and controls were 192.7 ± 13.9 ng/ml and 263.1 ± 22.4 ng/ml, respectively, and there was a statistically significant difference between the two groups (*p* < 0.05). We divided SCI patients into 4 groups according to their baseline serum Nogo-A quartile levels and analyzed their relationship with ASIA scores. The trend test results showed that with the increase of Nogo-A level, the ASIA sensation score and ASIA motor score were significantly decreased (*p* < 0.001). Multivariate regression analysis showed that serum Nogo-A levels remained a potential cause affecting the prognosis of SCI after adjusting for confounding factors in multiple models.

**Conclusions:**

Serum Nogo-A levels were significantly elevated in SCI patients. Moreover, elevated Nogo-A levels often indicate poor prognosis and can be used as a marker to predict the prognosis of SCI.

## 1. Introduction

The spinal cord injury (SCI) refers to damage to any part of the spinal cord or the nerve at the end of the spinal canal (cauda equina) that often results in permanent changes in strength, sensation, and other bodily functions below the injury site [1]. With the expansion of human activities in modern civilization, the incidence of SCI has gradually increased, with reported incidence ranging from 13/1 million to 220/1 million. Of these, developed countries have incidence rates of 13 to 163 per million people, while developing countries have rates ranging from 13 to 220 per million people [2]. SCI can be divided into traumatic SCI and nontraumatic SCI. A quick, traumatic impact to the spine that fractures, dislocates, pinches, or compresses one or more vertebrae can cause bleeding, edema, inflammation, and fluid buildup in and around the spinal cord, resulting in traumatic SCI [3, 4]. Arthritis, cancer, inflammation, infection, or degeneration of the spinal discs can all cause nontraumatic spinal cord injury. The socioeconomic burden of SCI is heavy. According to statistics, the annual cost of SCI in the United States is estimated to be between 5 million and 9 million US dollars, while in Australia, the figure is about 2 billion US dollars [5–7]. The pathogenic mechanism after SCI has not yet been fully elucidated, and the prognosis is poor, which affects the self-care ability of patients [8]. Therefore, finding prognostic markers for SCI and precise treatment are the top priorities.

Nogo-A, a membrane protein with a high molecular weight that is expressed on the surface of oligodendrocytes and neurons, is a growth inhibitory, antiadhesive, and growth cone collapse factor [9]. Nogo-A also has repellent and directing effects on growing neurites throughout development, influences the migration of early neural tube cells, and is a key limiting factor for axon regeneration and plasticity in the adult central nervous system [10]. In the adult and developing central nervous systems, Nogo-A is a key axonal development inhibitor. Nogo-A has been demonstrated to block neuronal and non-neuronal cell migration and spreading in vitro, which could have crucial consequences in CNS illnesses requiring angiogenesis, such as stroke, nerve injury, and retinal diseases [11, 12]. Nogo-A belongs to RTN4 family member, and its domain can interact with several different receptors, such as Nogo receptor 1 (NgR1) and immunoglobulin-like receptor (PirB) [13]. Although Nogo-A signals through different receptors, all of which converge to the Rho GTPase pathway, Nogo-A causes different effects.

In view of the neurite outgrowth inhibitory properties of Nogo-A, functional inhibitors of Nogo-A and its receptors have received extensive attention in spinal cord injuries in which axons cannot spontaneously regenerate. The purpose of our study is to observe the expression changes of Nogo-A and its relationship with prognosis in SCI patients, aiming to provide a new direction for the prevention and treatment of SCI.

## 2. Methods

### 2.1. Research Object

SCI patients admitted to Neck-Shoulder and Lumbocrural Pain Hospital of Shandong First Medical University since 2020 were screened. The patients who met the inclusion criteria but not the exclusion criteria were included in the study. Inclusion criteria were acute patients within 24 years of onset of SCI and consent to participate in this research. Exclusion criteria are as follows: age <18 years old or >80 years old; previous history of SCI; combined with severe heart, liver, lung, and kidney disease, etc.; combined with tumor or active immune disease; refused to participate in the study or did not cooperate with follow-up; and died within 3 months. Additionally, we recruited 52 volunteers to join the study as controls. The study was approved by the hospital ethics committee, and patients or family members gave full informed and written consent to the study.

### 2.2. Baseline Clinical Information

Baseline clinical information was collected after participants were enrolled. Information on age, gender, smoking, and alcohol consumption was collected through questionnaires. Data on blood pressure, blood glucose, leukocytes, and C-reactive protein were obtained from routine clinical hematology tests. All baseline clinical information was recorded by team members.

### 2.3. Serum Nogo-A Detection

Peripheral fasting venous blood was collected from all participants within 24 days of enrollment. Peripheral venous blood was left standing at room temperature for 20 minutes and then centrifuged in a low-temperature ultracentrifuge at a centrifugal speed of 12,000 g for a total of 10 minutes. After centrifugation, serum was collected and aliquoted into a -80 °C refrigerator [14, 15]. Reagents for the detection of Nogo-A were purchased from MyBioSource (San Diego, CA, USA), and all ELISA procedures were performed according to the instructions.

### 2.4. ASIA Scale Evaluation

The ASIA scale, developed by the American Spinal Cord Injury Association, is a general classification tool for spinal cord injury based on standardized sensory and motor assessments. This impairment scale includes motor and sensory examinations to determine left and right sensory and motor levels and overall neurological levels. In the ASIA sensory test, it is a clinical examination of 28 dermatomes to test whether sensation is absent (score of 0), impaired (score of 1), or normal (score of 2), with a total score of 224, with higher scores indicating that the sensory function is better. In the ASIA motor function test, scoring is based on evaluating 10 key upper and lower extremity muscles (score: 0-5). The total score of the ASIA motor score is 100, with higher scores indicating better motor function. The ASIA scale evaluation was completed by two trained physicians.

### 2.5. Statistical Analysis

Continuous variables and non-continuous variables were expressed as mean ± standard deviation or *n*, respectively, and *t*-test or chi-square analysis was used to further analyze differences between groups. The P for trend test was used to analyze the relationship between ASIA scale scores and Nogo-A interquartile range. Multivariate regression to explore the etiology that affects the prognosis of motor and sensory function in patients with SCI. SPSS 22.0 was used for statistical analysis, and the threshold for statistical difference was set at 0.05.

## 3. Results

### 3.1. Baseline Clinical Information

Baseline clinical information of SCI patients was counted. Clinical baseline information included age, gender, smoking, alcohol, systolic blood pressure (SBP), diastolic blood pressure (DBP), fasting blood glucose, leukocytes, and C-reactive protein. The statistical results are shown in Table 1. There was no statistically significant difference in baseline clinical information between the SCI group and the control group (*p* > 0.05).

### 3.2. ELISA Results

ELISA was used to detect serum Nogo-A levels. The baseline serum Nogo-A levels of SCI patients and controls were 192.7 ± 13.9 ng/ml and 263.1 ± 22.4 ng/ml, respectively, and there was a statistically significant difference between the two groups (*p* < 0.05). The specific results are shown in Table 1 and Figure 1.

### 3.3. Correlation between Serum Nogo-A and ASIA Score

We divided SCI patients into four groups according to the quartile range of serum Nogo-A levels and analyzed the ASIA sensory and motor function scores of each group. P for trend test was used to analyze the correlation between serum Nogo-A level and ASIA score. The results showed that both the ASIA sensory function score and the ASIA motor function score showed a downward trend with the increase of serum Nogo-A levels. The correlation analysis between the quartile levels of serum Nogo-A and the ASIA score is shown in Table 2.

### 3.4. Multivariate Regression Analysis

We performed multivariate regression analysis with ASIA functional function score and ASIA motor function score as dependent variables. The results showed that the serum Nogo-A score remained the etiological predictor of SCI prognosis in multiple adjusted models. The specific results of the multivariate regression analysis are shown in Table 3.

## 4. Discussions

The main finding of this study was that serum Nogo-A levels were significantly elevated in SCI patients, and elevated Nogo-A levels were associated with lower ASIA sensory and motor function scores. Through further regression analysis, it was found that the serum Nogo-A may be used as a biomarker for predicting the prognosis of SCI. Our study is the first to investigate the relationship between serum Nogo-A levels and prognosis of sensory and motor function in SCI patients.

Nogo, also known as a neurite outgrowth inhibitor or Reticulon 4, is a human protein that is mainly expressed by neurons during neural development and provides inhibitory signals for the migration and sprouting of central nervous endothelial cells. It has been identified as a CNS-specific inhibitor of neurite outgrowth [16]. RTN4 gene belongs to the reticular coding gene family and is involved in neuroendocrine secretion or membrane transport of neuroendocrine cells, and its product is a potent neurite outgrowth inhibitor [17, 18]. Additionally, three Nogo isomers have been identified: Nogo A, B, and c. Nogo-A, the most studied isoform, has two known inhibitory domains, including the N-terminal amino-Nogo and Nogo-66, which constitute extracellular loop molecules and are involved in the inhibition of nerve regeneration [19]. Among them, N-terminal amino-Nogo mainly inhibited neurite outgrowth, while Nogo-66 mainly caused growth cone destruction [20].

Nogo-A is involved in the pathogenesis of various neurological disorders. The study of Joseph et al. found that the expression of Nogo-A was significantly increased in rats with cerebral infarction; thus, its excitotoxicity and inhibitory effect on nerve regeneration may be one of the mechanisms of brain injury after cerebral infarction, and anti-Nogo-A treatment may be a potential avenue for the treatment of stroke [21]. A recent study by Rust et al. used a stroke model in mice with Nogo-A or its receptor S1PR2 gene deletion and found that it could improve the regeneration and repair of blood vessels after cerebral ischemia in mice and reduce neurological deficits, suggesting that the anti-Nogo-A treatment can improve the repair of blood vessels and nerves after ischemic central nerve injury [22]. As we all know, there is currently no effective treatment for ischemic stroke except thrombolysis [23]. In addition to the above two studies, the involvement of Nogo-A in ischemic stroke has been widely reported [24–27]. In addition to ischemic stroke, Chinese scholars have found that Nogo-A/PirB/TrkB pathway plays an inhibitory role in a rat model of intracranial hemorrhage, indicating that Nogo-A is involved in the pathogenic mechanism of secondary brain injury after intracerebral hemorrhage [28]. However, Japanese scholars found that in the rat model of intracranial hemorrhage, exercise training did not change the expression of Nogo-A in the brain, indicating that the role of Nogo-A in the rehabilitation of intracranial hemorrhage may be controversial, and further research is needed in the future [29]. Research from Xiangya Medical University shows that *α*-tocopherol has a neuroprotective effect on traumatic brain injury rats, and the mechanism may be that *α*-tocopherol can reduce the expression of Nogo-A and NgR in brain tissue after traumatic brain injury and promote the Neurodegeneration [30]. Another study from Shanghai Jiao Tong University found that in traumatic brain injury, elevated serum Nogo-A levels were strongly associated with poor prognosis, suggesting that Nogo-A levels could be used as a biomarker for predicting the prognosis of traumatic brain injury [31]. In addition, the role of Nogo-A in multiple sclerosis and immune encephalomyelitis has also been reported [32–34].

The role of Nogo-A in SCI has also attracted the attention of researchers. Swedish researchers found that Nogo-A knockout rats exhibited stronger neurodegenerative and neuroplasticity responses after SCI, suggesting that anti-Nogo-A therapy may be a new target for the treatment of SCI [35]. Swedish scholars further found that intrathecal anti-Nogo-A treatment can improve the regeneration and remodeling of the damaged central nervous system without obvious side effects [36]. The study by William B. J. Cafferty's team found that the synergistic effect of Nogo-A with MAG and OMgp is an important mechanism for inhibiting axonal regrowth and neural recovery after SCI [37]. For the first time, a multinational research team has demonstrated the efficacy of intra-tunnel injection of anti-Nogo-A antibodies in SCI patients [38]. Nevertheless, the research on the correlation between Nogo-A and SCI prognosis is still blank.

Our study has limitations. First, our sample size was not very large; second, we did not do longer-term follow-up; and finally, we did not do intervention studies. Nonetheless, we are the first report to investigate Nogo-A and prognosis in SCI.

## 5. Conclusions

Our study found that the serum Nogo-A level in SCI patients was higher than that in the normal population and was closely related to the degree of SCI injury. The serum Nogo-A may be one of the indicators to predict the degree of sensory and motor function recovery after SCI. This conclusion needs to be further confirmed and provide a new reference for the early intervention and intervention of SCI.

## Figures and Tables

**Figure 1:** Comparison of serum Nogo-A levels between the two groups. ∗*p* < 0.05 compared to controls. SCI, spinal cord injury.

**Table 1:** The clinical information of all participants.

	Controls (*n* = 52)	SCI (*n* = 108)	*p*
Age, years	53.1 ± 6.2	53.5 ± 6.7	0.718
Gender, male, *n* (%)	35 (67.3)	78 (72.2)	0.523
Smoking, *n* (%)	21 (40.4)	45 (41.7)	0.877
Drinking, *n* (%)	24 (46.2)	49 (45.4)	0.926
SBP, mmHg	113.3 ± 9.5	112.9 ± 9.2	0.799
DBP, mmHg	77.0 ± 5.8	77.3 ± 6.3	0.773
Fasting blood glucose, mmol/L	5.4 ± 0.6	5.6 ± 0.8	0.112
WBC, 10^9^/L	6.9 ± 1.3	7.3 ± 1.5	0.101
CRP, *μ*g/ml	4.1 ± 0.4	4.0 ± 0.5	0.209
Nogo-A, ng/ml	192.7 ± 13.9	263.1 ± 22.4	<0.001

Abbreviations: SCI, spinal cord injury; SBP: systolic blood pressure; DBP: diastolic blood pressure; WBC, white blood cells; CRP, C-reactive protein.

**Table 2:** Correlation between serum Nogo-A levels and SCI.

Variable	Serum Nogo-A levels (ug/ml)				*p*
	Q1	Q2	Q3	Q4	
ASIA sensation score	151.6 ± 17.1	144.9 ± 15.6	135.4 ± 13.2	124.1 ± 11.9	<0.001
ASIA motor score	83.1 ± 7.8	74.6 ± 6.5	66.2 ± 5.6	57.3 ± 4.8	<0.001

Abbreviations: SCI, spinal cord injury; ASIA, American Spinal Injury Association.

**Table 3:** Regression analysis of serum Nogo-A levels and ASIA scores.

	ASIA sensation score		ASIA motor score	
	Regression coefficient	*p* Values	Regression coefficient	*p* Values
Model 1	0.374	<0.001	0.368	<0.001
Model 2	0.283	<0.001	0.295	0.027
Model 3	0.246	0.033	0.251	0.042

Model 1: adjusted for age and gender; Model 2: further adjusted for smoking and drinking; Model 3: further adjusted for SBP, DBP, fasting blood glucose, WBC, and CRP. Abbreviations: ASIA, American Spinal Injury Association; SBP: systolic blood pressure; DBP: diastolic blood pressure; WBC, white blood cells; CRP, C-reactive protein.

## Data Availability

The study data presented may be made available from the corresponding author upon reasonable request.
